The article "miR-141-3p Targeted SIRT1 to Inhibit Osteogenic Differentiation of Bone Marrow Mesenchymal Stem Cells" was retracted in 2024. Reasons: signs of a paper mill; suspected computer-generated content; unreliable results or conclusions; concerns about the data.

# miR-141-3p Targeted SIRT1 to Inhibit Osteogenic Differentiation of Bone Marrow Mesenchymal Stem Cells

**DOI:** 10.1155/2023/9094092

**Published:** 2023-02-03

**Authors:** Shuzuo Zhou, Gang Zhang, Kun Wang, Zhong Yang, Yinghui Tan

**Affiliations:** Department of Stomatology, Second Affiliated Hospital of Army Military Medical University (Xin Qiao Hospital), Chongqing City 400038, China

## Abstract

**Purpose:**

To explore the expression of miR-141-3p during the osteogenic differentiation of human bone marrow mesenchymal stem cells (BMSCs) and its regulatory effect.

**Methods:**

Differentiation of BMSCs was induced by dexamethasone. The mRNA expression of miR-141-3p, ALP, RUNX2, and OCN was measured using RT-qPCR. The protein expression was detected via western blot. The target of miR-141-3p was predicted through the TargetScan website and confirmed using luciferase reporter assay.

**Results:**

miR-141-3p expression declined during osteogenic differentiation. The relative ALP activities and the mRNA expression of ALP, RUNX2, and OCN were markedly reduced in the miR-141-3p mimic group while increased in the inhibitor group. Cell viability was suppressed in the miR-141-3p mimic group and promoted in the inhibitor group. SIRT1 was predicted to be a downstream gene of miR-141-3p, and this prediction was confirmed via the luciferase reporter assay. The results of the western blot assay demonstrated that SIRT1 expression was decreased in the miR-141-3p mimic group. SIRT1 reversed the inhibitory influence of miR-141-3p on the osteogenic differentiation ability of BMSCs.

**Conclusion:**

miR-141-3p targeted SIRT1 to inhibit osteogenic differentiation of BMSCs via the Wnt/*β*-catenin signaling pathway.

## 1. Introduction

Periodontal disease is the first high incidence disease of the human oral cavity. Under the long-term continuous inflammation stimulation, the alveolar bone can undergo pathological absorption and eventually lead to tooth loosening or even loss [1, 2]. With the deepening of tissue-engineering research, the role of stem cells in bone tissue repair is increasingly prominent [3, 4], but limitations such as limited in vitro amplification capacity, complex biological effects, and major biological functions which can be replaced by bioactive molecular combinations hinder the development and application [5, 6].

BMSCs are a kind of pluripotent stem cells with self-renewal ability [7]. BMSCs can be cultured in vitro and induced into osteoblasts, chondroblasts, adipocytes, and other cell types by different induction solutions [8]. Differentiation of BMSCs into osteoblasts is essential in maintaining normal bone stability and is an important target for the research of bone metabolism drugs [9]. Therefore, elucidating the mechanism of osteogenic differentiation of BMMSCs and changing the differentiation direction of BMSCs are potential methods to treat osteoporosis in the future.

Recent studies have found that miRNAs could regulate the differentiation of osteogenic cells such as bone marrow mesenchymal stem cells (BMSCs) and affect the process of bone tissue generation and resorption [10]. The human coding genes regulated by miRNAs account for 40%-90% of the total [11] and widely affect cell proliferation, differentiation, and apoptosis and the progress of cardiovascular diseases, neurodegenerative diseases, tumors, and other diseases [10]. Studies have shown that changes in miRNA will have an obvious impact on the function of BMSCs [12]. miRNAs participate in biological processes by regulating target genes and are essential in the pathogenesis of bone development and pathogenesis of osteoporosis [13–15]. For example, miR-9 and miR-133 could inhibit the osteogenic differentiation of BMSCs via inhibiting Runx2 [16]. miR-302a enhances osteogenic differentiation of mouse embryonic precursor cells through inhibiting the expression of COUP-TFII [17]. However, miR-141-3p is poorly studied in the osteogenic differentiation of BMSCs. Exploring the role of miR-141-3p and its relation with the target in BMSCs would improve the current understanding of the mechanisms underlying the osteogenic differentiation of BMSCs.

This study verified the expression of miR-141-3p during osteogenic differentiation *in vitro* experiments, observed its effect on osteogenic differentiation, and confirmed its regulatory effect on the putative target gene SIRT1.

## 2. Methods

### 2.1. Cell Culture and Osteogenic Differentiation

BMSCs obtained from the American Type Culture Collection (ATCC; Manassas, USA) were cultured with the *α*-MEM cell culture medium in a 37°C constant temperature incubator containing 5% CO_2_. When the cells almost covered the bottom, 0.25% trypsin was added for digestion and passage. After BMSCs were cultured for 24 h under normal conditions, BMSCs were added with 10% fetal bovine serum, 0.2 mmol/l ascorbic acid, 1% glutamine, 10 nmol/l dexamethasone, and 10 mmol/l *β*-glycerophosphate to induce osteogenic differentiation. BMSCs were induced and cultured in DMEM for 21 days.

### 2.2. Measurement of Alkaline Phosphatase Activity (ALP)

ALP viability was detected using a commercial kit. Cell lysates were added to a freshly prepared substrate with an alkaline phosphatase kit and cultured for 30 min before NaOH was used as a stop. The absorbance at 405 nm was measured. After two washes with PBS, the collected cells were fixed for 10 min and cultured in the dark environment using a BCIP/NBT reagent for 30 min before ALP staining.

### 2.3. RT-qPCR Assay

Using TRIzol, total RNA was extracted. The RNA was then reverse transcribed using the reverse transcription kit. The mRNA expression levels of miR-141-3p and SIRT1 were evaluated through the 2^-△△CT^ method. The primer sequence is shown in Table 1.

### 2.4. Western Blot

Cells were lysed on ice using the RIPA lysate (Cell Signaling Technology, USA). After the steps of protein extraction, protein concentration determination, electrophoresis, membrane transfer, and sealing, the primary antibody (Abcam, UK) was added and incubated overnight at 4°C. Then, the secondary antibodies (Abcam, UK) were added and incubated for 2 h at 37°C. The relative expression of proteins was detected using a chemiluminescence gel imaging system.

### 2.5. CCK-8 Assay

3 × 10^4^ transfected cells in each group were seeded in a 96-well plate, then maintained in 10 *μ*l CCK-8 reagent (Thermo Fisher, USA) at 0 h, 24 h, 48 h, and 96 h and at 37°C before color development. The absorbance (OD) value was detected at 450 nm.

### 2.6. Luciferase Reporter Assay

The SIRT1 wild-type plasmid and the SIRT1 mutant plasmid were constructed. miR-224 mimic/negative control and SIRT1-WT or SIRT1-MUT were cotransfected using Lipofectamine 2000. The luciferase activity was evaluated via a dual-luciferase activity assay kit (Promega, USA) after 48 h.

### 2.7. Statistical Analysis

Statistical analysis was conducted with SPSS 21.0. Comparison between groups was conducted with one-way ANOVA. *P* < 0.05 suggested significant differences.

## 3. Results

### 3.1. The miR-141-3p Expression Was Decreased during Osteogenic Differentiation

After osteogenic induction for 21 d, the relative ALP activity was obviously raised (Figure 1(a)). miR-141-3p was more highly expressed in osteoporotic samples (Figure 1(b)). miR-141-3p expression declined during osteogenic differentiation (Figure 1(c)). The mRNA expression (Figure 1(d)) and protein expression (Figure 1(e)) of SIRT1 were raised during osteogenic differentiation.

### 3.2. The miR-141-3p Suppressed the Osteogenic Differentiation Ability of BMSCs

The miR-141-3p mimic obviously raised the miR-141-3p expression while the inhibitor observably decreased it (Figure 2(a)). Cell viability was suppressed in the mimic group and promoted in the inhibitor group (Figure 2(b)). The relative ALP activities were suppressed in the mimic group while raised in the inhibitor group (Figure 2(c)). In addition, the mRNA expression of ALP (Figure 2(d)), RUNX2 (Figure 2(e)), and OCN (Figure 2(f)), which were osteogenic transcription factors, was suppressed in the mimic group and raised in the inhibitor group.

### 3.3. SIRT1 Was Directly Regulated by miR-141-3p

The 3′UTR of SIRT1 mRNA is partially complementary to the miR-141-3p sequence as predicted by the website (Figure 3(a)). The luciferase activity of SIRT1-WT was suppressed by the miR-141-3p mimic (Figure 3(b)). Furthermore, SIRT1 expression was inhibited in the miR-141-3p mimic group while enhanced in the miR-141-3p inhibitor group (Figure 3(c)).

### 3.4. SIRT1 Reversed the Detraction Influence of miR-141-3p on Osteogenic Differentiation of BMSCs

SIRT1 expression declined in the miR-141-3p mimic group while oe-SIRT1 increased it (Figure 4(a)). Cell viability was repressed in the miR-141-3p mimic group, but overexpressed SIRT1 reversed this effect (Figure 4(b)). The relative ALP activities were repressed in the miR-141-3p mimic group, but overexpressed SIRT1 reversed this effect (Figure 4(c)). In addition, the mRNA expression of ALP (Figure 4(d)), RUNX2 (Figure 4(e)), and OCN (Figure 4(f)) was repressed in the miR-141-3p mimic group while overexpressed SIRT1 reversed this effect.

### 3.5. miR-141-3p Suppressed Wnt/*β*-Catenin Signaling Pathway to Inhibit Osteogenesis

miR-141-3p mimic obviously repressed the expression of *β*-catenin, Bcl-2, and Cyclin D1 while overexpressed SIRT1 reversed this effect (Figure 5).

## 4. Discussion

The periodontal tissue destruction caused by periodontal disease is related to the immune inflammatory response caused by pathogenic bacteria, and various inflammatory factors in periodontitis can lead to progressive osteolysis and inhibit bone formation [18]. Bone homeostasis refers to the balance between osteoblast-dominated bone formation, which is mainly controlled by the differentiation of BMSCs into osteoblast-dominated series of cells [9]. BMSCs are a class of stem cells with multidirectional differentiation potential and could be differentiated into osteoblasts under specific environments and regulate the growth and development of the bone [8]. Because BMSCs have the characteristics of wide sources, easy separation and culture, and great differentiation potential, they are considered as the ideal cell for treating bone tissue damage and bone regeneration repair. However, how to enable unidirectional osteogenic differentiation of BMSCs is critical to restrict the efficiency of clinical repair. miRNA could bind to the 3′UTR region of related genes to suppress its translation and then affect numerous biological processes [10, 19]. Studies have confirmed that miRNAs are essential in BMSC osteogenic differentiation [20, 21]. For example, in osteogenic differentiation, RUNX2 is a targeted regulatory gene of miR-135 [22]. miR-214 inhibits osteogenic differentiation by targeting Osterix [23].

miR-141-3p is located at chromosome 12pl3.31 [24]. miR-141-3p could change the cellular biological processes through the regulation of different target genes or signaling pathways [25]. miR-141-3p is differently expressed in different human tumors [26]. This study suggested that the miR-141-3p expression was decreased during osteogenic differentiation. OCN and RUNX2 are the hallmark proteins of osteogenic differentiation, and ALP activity is a quantitative measure reflecting both osteogenic activity and osteogenic capacity. miR-141-3p mimic repressed the relative ALP activities; the mRNA expression of ALP, RUNX2, and OCN; and cell viability. The miR-141-3p inhibitor showed the opposite effect. Thus, it can be seen that miR-141-3p was essential in osteogenic differentiation.

The regulatory network of genes in the body is a huge and complex process. The miRNA can regulate target genes to participate in the physiological process of cells. Anderson and McAlinden found that miR-483 could target Smad4 to inhibit human BMSC (hBMSC) differentiation into chondrocytes [27]. Zhang et al. found that miR-146b-5p promoted the neural transformation of pluripotent stem cells via regulating the target gene [28]. SIRT1 was guessed to be downstream of miR-141-3p, and the luciferase reporter assay confirmed this prediction. SIRT1 was lower expressed under the miR-141-3p mimic. The inhibitory effect of miR-141-3p on osteogenic differentiation was reversed by SIRT1. Thus, it can be seen that miR-141-3p suppressed osteogenic differentiation of BMSCs via downregulated SIRT1. SIRT1 is essential in bone metabolism, but the specific mechanism is still being studied. SIRT1 expression was significantly decreased in the femoral neck of OP patients, and SIRT1 activity in peripheral blood mononuclear cells was also decreased, indicating that there was a close relationship between SIRT1 and OP [29]. SIRT1 can improve postmenopausal osteoporosis by downregulating SOST in vivo and can also improve postmenopausal osteoporosis and reverse abnormal bone mineralization [30].

It was found in the in vitro study that the increased expression of SIRT1 promoted the expression of SOX9 and RUNX2, and the acetylation level of catenin was significantly reduced [31]. After inhibiting Wnt/*β*-catenin signaling, markers of osteogenic differentiation of BMSCs were significantly decreased, indicating that SIRT1 can promote bone formation via activating the Wnt/*β*-catenin pathway [32], which is a classical pathway of bone metabolism [33]. The miR-139-5p downregulated the CTNNB1 and FZD4 expression through the Wnt/*β*-catenin pathway, thereby inhibiting osteogenic differentiation of BMSCs [34]. Overexpressed lncRNA HULC enhanced the activation of the Wnt/*β*-catenin signaling pathway by downregulating miR-195, subsequently promoting osteogenic differentiation [35]. This suggested that the miRNA-mediated Wnt/*β*-catenin signaling pathway is essential in BMSC osteoblast differentiation. Similarly, we found that miR-141-3p suppressed the Wnt/*β*-catenin signaling pathway to repress osteogenesis.

This study has some limitations. This study only found the effect of miR-141-3p during the osteogenic differentiation of BMSCs and its regulatory effect in vitro. But there is no evidence of in vivo experiments. Further study in vivo is needed.

In conclusion, miR-141-3p targeted SIRT1 to inhibit osteogenic differentiation of BMSCs through the Wnt/*β*-catenin pathway.

## Figures and Tables

**Figure 1:** miR-141-3p was downregulated during osteogenic differentiation. (a) ALP activities were evaluated by spectrophotometry. (b, c) The miR-141-3p expression in osteoporotic samples (b) and BMSC-induced osteogenic differentiation (c) was measured via RT-qPCR. (d) The mRNA expression of SIRT1 was evaluated. (e) Protein expression of SIRT1 was examined using western blot. ^∗^*P* < 0.05.

**Figure 2:** The miR-141-3p suppressed the osteogenic differentiation ability of BMSCs. (a) The miR-141-3p expression was examined via RT-qPCR. (b) CCK-8 assay was applied to evaluate cell viability. (c) ALP activities were evaluated by spectrophotometry. (d) The mRNA expression of ALP, (e) RUNX2, and (f) OCN was examined via RT-qPCR.

**Figure 3:** miR-141-3p regulates SIRT1 expression via targeting its 3′UTR. (a) The predicted binding sites. (b) Inhibiting effect of miR-141-3p mimic on luciferase activity of SIRT1-WT. (c) The miR-141-3p regulated SIRT1 protein level. ^∗^*P* < 0.05.

**Figure 4:** SIRT1 reversed the inhibitory influence of miR-141-3p on osteogenic differentiation ability of BMSCs. (a) miR-141-3p expression was examined. (b) CCK-8 assay was done to observe cell viability. (c) ALP activities were evaluated by spectrophotometry. (d) The mRNA expression (e) RUNX2, and (f) OCN were examined via RT-qPCR.

**Figure 5:** miR-141-3p suppressed Wnt/*β*-catenin signaling pathway to inhibit osteogenesis. ^∗^*P* < 0.05.

**Table 1:** Primer sequence.

Target	Primer sequence(5′-3′)
miR-141-3p	F:GCGGAAAGAGGCCCCG
	R:AGTGCAGGGTCCGAGGTATT
U6	F:CTCGCTTCGGCAGCACA
	R:AACGCTTCACGAATTTGCGT
SIRT1	F: TGCCGGAAACAATACCTCCA
	R:AGACACCCCAGCTCCAGTTA
*β*-Actin	F:ACGTCACGAACTACTAGCAAT
	R:TGTGTGCATGAGTCTCTCCACG

## Data Availability

Data to support the findings of this study is available on reasonable request from the corresponding author.
